The article "A Deep Neural Network Ensemble Classifier with Focal Loss for Automatic Arrhythmia Classification" was published in 2022. Journal: J Healthc Eng.

# A Deep Neural Network Ensemble Classifier with Focal Loss for Automatic Arrhythmia Classification

**DOI:** 10.1155/2022/9370517

**Published:** 2022-09-09

**Authors:** Han Wu, Senhao Zhang, Benkun Bao, Jiuqiang Li, Yingying Zhang, Donghai Qiu, Hongbo Yang

**Affiliations:** ^1^School of Biomedical Engineering (Suzhou), Division of Life Science and Medicine, University of Science and Technology of China, Hefei 230026, China; ^2^Suzhou Institute of Biomedical Engineering and Technology, Chinese Academy of Science, Suzhou 215163, China

## Abstract

Automated electrocardiogram classification techniques play an important role in assisting physicians in diagnosing arrhythmia. Among these, the automatic classification of single-lead heartbeats has received wider attention due to the urgent need for portable ECG monitoring devices. Although many heartbeat classification studies performed well in intrapatient assessment, they do not perform as well in interpatient assessment. In particular, for supraventricular ectopic heartbeats (S), most models do not classify them well. To solve these challenges, this article provides an automated arrhythmia classification algorithm. There are three key components of the algorithm. First, a new heartbeat segmentation method is used, which improves the algorithm's capacity to classify S substantially. Second, to overcome the problems created by data imbalance, a combination of traditional sampling and focal loss is applied. Finally, using the interpatient evaluation paradigm, a deep convolutional neural network ensemble classifier is built to perform classification validation. The experimental results show that the overall accuracy of the method is 91.89%, the sensitivity is 85.37%, the positive productivity is 59.51%, and the specificity is 93.15%. In particular, for the supraventricular ectopic heartbeat(s), the method achieved a sensitivity of 80.23%, a positivity of 49.40%, and a specificity of 96.85%, exceeding most existing studies. Even without any manually extracted features or heartbeat preprocessing, the technique achieved high classification performance in the interpatient assessment paradigm.

## 1. Introduction

An electrocardiogram is a sequence that records the electrical activity of the heart [1]. With the increase in the number of heart diseases [2] and the rapid development of computer technology such as deep learning, there is a growing interest in how to use computer technology to aid in the automatic diagnosis of heart diseases [3, 4]. The automated diagnosis of arrhythmias, one of the most common cardiac diseases, has been a popular area of research in computer-aided diagnosis [5]. It consists of two main challenges. The first is the dataset's high imbalance, with normal beats taking up the majority of the ECG signal. The normal beats (N) account for more than 90% of all beats in the MIT-BIH arrhythmia dataset. Second, the training and testing sets used in the interpatient evaluation paradigm are from different populations, which is more in line with our actual requirements for automatic arrhythmia diagnosis, but the prediction difficulty is greatly increased due to individual variability of different populations.

The article "A Deep Neural Network Ensemble Classifier with Focal Loss for Automatic Arrhythmia Classification" was published in 2022. Journal: J Healthc Eng.

The existing arrhythmia classification algorithms include two main types, depending on the input data. The one is arrhythmia classification based on manual feature extraction, and the other is arrhythmia classification based on automatic feature extraction [5].

In the method of manual feature extraction, the manually extracted features [3, 6, 7, 8, 9, 10, 11, 12, 13, 14] mainly include RR interval, short-time Fourier transform, morphological features, empirical modal decomposition, higher-order statistics, and entropy metric. Then machine learning classifiers are adopted to classify the extracted features, including the weighted linear discriminator [15, 16, 17, 18], support vector machine [4, 19, 20, 21, 22, 23], multilayer perceptron [24], and convolutional neural network [25, 26, 27, 28]. Chazal et al. [29] extracted five groups of features, including R-R, HOS, wavelet, morphology, and LBP, from ECG signals and used these features to classify ECG signals by linear classifier. H. Shi et al. [30] extracted six groups of features, including RR interval, morphology, statistics, higher-order statistics, wavelet transform, and wavelet packet entropy, then used a hierarchical XGBoost classifier for classification. Dias et al. [31] manually extracted the RR interval, morphology features, and higher-order features of ECG signals and used an LD classifier to classify arrhythmia. Yang et al. [32] constructed a hybrid kernel-based extreme learning machine to compare different combinations of feature inputs, which yielded the best classification results when ten randomly selected combinations of feature inputs were used in the input. However, these methods rely excessively on manual feature selection, which increases the complexity of the computational process and the time required to extract features upfront.

With the rapid growth of deep learning, there is a need to use deep learning for automatic heartbeat classification by simply inputting the raw ECG data and then enabling the deep learning algorithm to learn the features for us and provide the final classification result [33, 34, 35]. Garcia et al. [36] explored a vector ECG-based deep convolutional neural network-based arrhythmia classification method to classify three beats, N, SVEB(S), and VEB(V). Takalo-Mattila et al. [37, 38] used a high-pass filter, band-stop filter, and low-pass filter to remove noise from the ECG signal, then sliced the ECG signal according to the location of the marked *R* peaks in the database, and finally used a convolutional neural network to classify the four beats of N, S, V, and F. Li et al. [39] used equal time (5 s) slicing of the raw ECG, the discrete wavelet transform for noise removal, and a deep residual convolutional neural network for classification. However, the sensitivity of S was often low in these studies, making it challenging to apply in real-life situations. Sellami et al. [40] used a robust deep convolutional network to classify arrhythmia. The authors created a batch-weighted loss function to alleviate the data imbalance problem and used three different heartbeat input patterns for experimental comparison. In the classification model, S had a high sensitivity, whereas N had a low sensitivity when compared to other algorithms. Niu et al. [41] used the SBCX method to process the input beats, effectively removing the effect of baseline drift noise. At the same time, the authors combined the processed heartbeat signal and RR interval features together as the input data for classification. The classification effect was good, but too much preprocessing was carried out, and the classification process was not automated enough.

The article "A Deep Neural Network Ensemble Classifier with Focal Loss for Automatic Arrhythmia Classification" was published in 2022. Journal: J Healthc Eng.

Based on these problems, this article proposes a new heartbeat segmentation method and constructs a deep neural network ensemble classifier with focal loss. It performs effective arrhythmia classification without any preprocessing using only raw heartbeat data.

We present the ECG dataset used and discuss the details of the implementation of the heartbeat classification algorithm in this article in the next section. In Section 3, we compare the algorithm suggested in this article to some existing algorithms and conduct ablation studies on the algorithm's primary components. We conclude this article in Section 4.

## 2. Methods

The overall structure diagram of the proposed classification system is shown in Figure 1. The publicly available MIT-BIH arrhythmia dataset is used as the input heartbeat in this article. After heartbeat sampling, the input heartbeat data are segmented using a special heartbeat segmentation method and used as the training set. The deep convolutional neural network ensemble classifier's training process uses focal loss as the loss function, and the classifier is voted to obtain the final classification results. The method proposed in this paper is validated under the interpatient assessment paradigm.

The article "A Deep Neural Network Ensemble Classifier with Focal Loss for Automatic Arrhythmia Classification" was published in 2022. Journal: J Healthc Eng.

### 2.1. ECG Database

The MIT-BIH arrhythmia database, which contains 48 30-minute long records from 47 patients, is used for the raw data. The dataset includes detailed annotations from cardiologists containing the type of heartbeat for each beat and the location of each *R*-peak peak [42].

For comparison, the ECG dataset is partitioned into DS1 and DS2, as described in [29]. In the interpatient evaluation paradigm, a modified limb lead II (MLII) is used to go as the input signal for the model, using DS1 for training and DS2 for experimental testing. As shown in Table 1, the heartbeat types are classified into five categories according to the American Association for the Advancement of Medical Devices (AAMI). Four records with rhythm are excluded, as suggested by AAMI. The specific division is shown in Table 2.

### 2.2. Segmentation of ECG Signals

Following the database division, each heartbeat record is segmented based on the R-peak annotation location provided by the dataset.  Table 3 shows the segmentation lengths of the different methods and the sensitivity of the S in the final classification results. It can be seen that most methods have a heartbeat segmentation length of 300 or less. Due to the high degree of similarity between S and N, and the small proportion of S in the overall heartbeats, it is easy to cause overfitting of S during the training process, resulting in low sensitivity of S. Under the interpatient assessment paradigm, Garcia (2017) and Takalo-Mattila (2018) had a classification sensitivity of just around 60% for S [36, 37]. Jinghao Niu (2020) and Haojie Zhang (2021) had higher sensitivity of S (77.35% and 88.24%), respectively, but their training data not only contained the original signal of the heartbeat but also included the manually extracted R-R interval features [39, 41]. After removing the R-R interval features, Haojie Zhang (2021) and Jinghao Niu (2020) both had extremely low sensitivity (38.7% and 8.06%).

In this article, we want the model to be able to classify heartbeats automatically using only the raw heartbeat signal, with no data preprocessing or manual feature input. So, we provide a new heartbeat segmentation strategy.  Figure 2 shows the difference between the traditional single heartbeat segmentation approach and the heartbeat segmentation approach in this article.  Figure 2(a) shows the traditional single heartbeat segmentation method [41].  Figure 2(b) shows the segmentation approach in this article. The length of the heartbeat window in this article is 508, consisting of 250 samples before and 257 samples after the R-peak.  Figure 2(c) shows a comparison of N and S in the two segmentation methods.  Figure 2(c)(i) and Figure 2(c)(ii) show the N segmented by the conventional 256 sampling points and the 508 sampling points segmentation of this article, respectively, while Figure 2(c)(iii) and Figure 2(c)(iv) show the S segmented by the conventional 256 sampling points and the 508 sampling points segmentation of this article, respectively. Comparing Figure 2(c)(i) and Figure 2(c)(iii), it can be seen that the morphology of N and S is highly similar in the traditional segmentation method, which makes it difficult for the classifier to distinguish N and S. Comparing Figure 2(c)(ii) and Figure 2(c)(iv), it can be seen that the segmentation method in this article increases the window length of the heartbeat, which is conducive to extracting more neighbourhood features from the original signal. The morphological distinctions between *N* and *S* are bigger when applying the segmentation method in this research, making it easier for the classifier to distinguish between the two.

The article "A Deep Neural Network Ensemble Classifier with Focal Loss for Automatic Arrhythmia Classification" was published in 2022. Journal: J Healthc Eng.

Table 4 shows the proportions of each class of heartbeats after segmentation. To make the classification more automated, this article does not apply any filtering to the segmented heartbeat signals and only inputs the raw heartbeat data for classification. The proportion of heartbeats following segmentation is severely unbalanced, as shown in Table 4. To prevent overfitting in the training, the effect of data imbalance needs to be further weakened.

### 2.3. Overall Structure of the Algorithm and Heartbeat Sampling

Figure 3 shows the general structure of the method. Based on the interpatient paradigm, the MIT-BIH arrhythmia database is classified into DS1 and DS2. Then, for N, random sampling is used, and incremental sampling is used for the remaining data classes [43]. The neural network is trained using the obtained samples from DS1. Six focal loss deep neural network classifiers are trained in total, and the final arrhythmia classification result is determined by voting on them.

Random sampling and incremental sampling in DS1 mitigate the effects of data imbalance. Unlike previous research [37, 39, 40, 41, 44], this publication raises the sampling size for class *S* to 7544, for class *V* to 4592, and for class *N* to be randomly sampled with a size of 11188 and the sizes of *F* and *Q* remain unchanged,.

There are two main reasons why such a unique approach to data sampling is chosen. Firstly, we want the classifier to focus more on the classification of *S*, so *S* accounts for the largest proportion of abnormal heartbeats in the training set. Secondly, the final result is a vote for each focal loss deep neural network classifier. In the training set of each classifier, only *N* is a random sample from DS1; the rest of the samples are the same. According to the theory of ensemble learning [45, 46], when the base classifiers have the same classification performance, the higher the independence of each base classifier, the better the overall classification performance. As a result, the highest percentage of *N* (47.11%) is found in each training set.

The article "A Deep Neural Network Ensemble Classifier with Focal Loss for Automatic Arrhythmia Classification" was published in 2022. Journal: J Healthc Eng.

### 2.4. Focal Loss Function

After random sampling and incremental sampling of DS1, the impact of data imbalance is mitigated. To further reduce the problem of overfitting, the focal loss function is adopted.

The focal loss was proposed by He et al. [47] to address the problem of difficult imbalance in classification among data in dense object detection. The amount of data containing objects in object detection is much smaller than the amount of data without objects, and the difficulty of classifying data without objects is low, which has a very small improvement effect on the model. Focal loss reduces the weight of easily classifiable samples, allowing the model to focus more on the hard-to-classify samples.

(1) $$\begin{array}{c} CE=-\log\left(P_{t}\right)\text{,} \end{array}$$

(2) $$\begin{array}{c} Lf=-a_{t}{\left(1-P_{t}\right)}^{y}\;\log\left(P_{t}\right)\text{.} \end{array}$$

In (1) and (2), *P*_*t*_ represents the probability of the predicted value. Equation (1) is the traditional cross-entropy loss function, where the closer *P*_*t*_ is to 1, the smaller the loss value (CE) is, thus achieving the training purpose by making the total loss value decrease in the training of the model. Equation (2) is the local loss function, compared to the traditional cross-entropy loss function added*a*_*t*_ and(1 − *P*_*t*_)^*y*^. The proportion of loss value weights for different samples can be adjusted by *a*_*t*_, which helps us to alleviate the problems caused by data imbalance. For (1 − *P*_*t*_)^*y*^, the proportion is smaller when *P*_*t*_ is closer to 1. Therefore, we can make the model pay more attention to data with smaller *P*_*t*_ values, thus increasing the model's attention to the hard-to-classify samples. In this study, such a focus is very important. We can adjust the size of *y* to make the model more focused on the distinction between *N* and *S*.

In this article, we choose *y* = 2.35 and use different weighting ratios for different heartbeat categories. The specific weight ratio is *N* : *S* : *V* : *F* : *Q* = 1.6 : 1.8 : 0.8 : 1.0 : 1.0.

### 2.5. Structure of the Deep Residual Convolutional Neural Network

Figure 4 shows the classification model structure for each base classifier. The target heartbeats and their category labels comprise the input data.

The article "A Deep Neural Network Ensemble Classifier with Focal Loss for Automatic Arrhythmia Classification" was published in 2022. Journal: J Healthc Eng.

The network consists of 9 convolutional layers, each with a convolutional kernel size of 17. The first five convolutional layers include 20 convolutional kernels, while the final four convolutional layers contain 40 convolutional kernels. A batch normalization [48] process is added after each convolutional layer to speed up the training process. The use of “Tanh” after the first convolutional layer and “ReLU” after the other convolutional layers allows the model to better adapt to the data. To prevent overfitting during the deep convolutional neural network training, a 40% dropout is added after 3–9 convolutional layers [49]. To enable the network to be trained at a deeper level, the residual structure proposed by Kaiming He et al. [50] is used. The addition of jump connections helps to weaken the problem of depth information loss. After the last jump connection, batch normalization and “ReLU” processing are again performed. Finally, our base classifier results are obtained after global average pooling and a fully connected layer.

## 3. Results and Discussion

### 3.1. Performance Metrics

To evaluate the performance of the model, the confusion matrix of the model is given, and four statistical performance metrics are adopted to evaluate our method as a whole according to the guidelines provided by AAMI [29], namely, accuracy (Acc), sensitivity (Sen), positive productivity (+P), and specificity (Spe). The calculation of each metric is defined in the following equations:

(3) $$\begin{array}{c} Acc\left(\%\right)=\frac{TP+TN}{TP+FP+TN+FN}\times 100\%\text{,} \end{array}$$

(4) $$\begin{array}{c} Sen\left(\%\right)=\frac{TP}{TP+FN}\times 100\%\text{,} \end{array}$$

(5) $$\begin{array}{c} +P\left(\%\right)=\frac{TP}{TP+FP}\times 100\%\text{,} \end{array}$$

(6) $$\begin{array}{c} Spe\left(\%\right)=\frac{TN}{TN+FP}\times 100\%\text{.} \end{array}$$

When calculating the overall model performance metric, TP is defined as the number of correctly classified abnormal heartbeats, TN is defined as the number of normally classified normal heartbeats, FP indicates the number of normal heartbeats classified as abnormal, and FN indicates the number of abnormal signals classified as normal.

### 3.2. Experimental Results and Discussion

The model performance for the six base classifiers and the final ensemble classifier is shown in Table 5. The overall accuracy (Acc) of the base classifiers is all above 83%, with the majority exceeding 88%. Most of the sensitivities (Sen) are around 85%. The final classification result is obtained after voting for the six base classifiers.

As shown in Table 5, the final ensemble classification results are significantly better than the average metrics of all six classifiers. Accuracy (Acc) increases by 4.26% (87.63% to 91.89%), positive productivity (+P) increases by 12.75% (46.76% to 59.51%), sensitivity increases by 1.18% (84.19% to 85.37%), and specificity (Spe) increases by 4.34% (88.81% to 93.15%). The accuracy (Acc) of the 6th base classifier is low in Table 5. There are two reasons for this. First, neural network training has a chance. Second, in the focal loss function in this article, S has a high weight, which may cause the classifier to overfocus on S during the training process. The confusion matrix of the final classification results is given in Table 6.

The article "A Deep Neural Network Ensemble Classifier with Focal Loss for Automatic Arrhythmia Classification" was published in 2022. Journal: J Healthc Eng.

Table 7 shows the sensitivity (Sen), positive productivity (+P), and specificity (Spe) for classes N, S, and V and compares them with six classical arrhythmia classification algorithms.  Table 8 shows the overall performance of the model in terms of accuracy (Acc), positive productivity (+P), sensitivity (Sen), and specificity (Spe) and compares it with the classical algorithms.

In Tables 7 and 8, the model input data for Garcia (2017), Takalo-Mattila (2018), Sellami (2019), and Yuanlu Li (2021) are all raw heartbeat signals without the inclusion of manually extracted heartbeat features [36, 37, 39, 40].

Among them, the accuracy of Garcia (2017) is slightly higher than the method proposed in this article (92.38% to 91.89%), and the sensitivity of N is also slightly higher than that of the method proposed in this article (93.99% to 93.15%). However, the sensitivity of S in this article is much higher than that of Garcia (2017) (80.23% to 61.96%). The sensitivity of V in this article is slightly higher than that of Garcia (2017) (90.99% to 87.34%) and the productivity (+P) of V is much higher than that of Garcia (2017) (83.09% to 59.44%). Of interest is that Garcia (2017) only achieved 3 classifications, rounding off F and *Q* in the training process, whereas this article is the result of 5 classifications, which is much more difficult. The recognition of abnormal heartbeats is especially significant in classifying arrhythmia, which is related to the model's effectiveness in real-world applications. Reflecting on the overall metrics of the model, in Table 8, the sensitivity (Sen) of the algorithm in this article is higher than it (85.37% to 81.73%). Thus, although the method proposed in this article is slightly lower in terms of overall accuracy (Acc), the model is more effective in practical applications [36].

Takalo-Mattila (2018) used a convolutional neural network with three convolutional layers to classify the heartbeat signal. Although the adoption of a smaller network structure to perform classification is advantageous in terms of reducing training time, it has a significantly lower classification effect than the approach in this study. Despite the model structure being more complex, our input heartbeats do not need to be denoised. This also reduces the overall time and better reflects the model's automation [37].

The article "A Deep Neural Network Ensemble Classifier with Focal Loss for Automatic Arrhythmia Classification" was published in 2022. Journal: J Healthc Eng.

The accuracy of the proposed algorithm is higher than that of Sellami (2019) (91.89% to 89.91%) and the sensitivity of N is higher than that of Sellami (2019) (93.15% to 88.52%). The sensitivity of S in this article is slightly lower than that of Sellami (2019) (80.23% to 82.04%), but the productivity (+P) is higher than it (49.40% to 30.44%). The sensitivity of V in this article is slightly lower than that of Sellami (2019) (90.99% to 92.05%), but the productivity (+P) is higher (83.09% to 72.13%). Sellami (2019) has a high classification performance for all types of heartbeats. However, it has a slightly lower sensitivity to N of only 88.52% compared to other methods. The algorithm in this article has comparable classification results for S and V but has a higher sensitivity to N(93.15%) [40].

Yuanlu Li (2021) desired a more automated classification algorithm and therefore used an equal-length segmentation method that did not require R-peak location. However, the sensitivity of S in their classification results is too low, at only 35.22%. This causes its classification model to almost fail in identifying S. In Table 8, the overall sensitivity of their model is the lowest at just 52.10%, making it difficult to apply in real-life situations [39].

De Chazal (2004) and Jinghao Niu (2020) used manually extracted features in their input data. De Chazal (2004) extracted many domain-specific features from the two-lead ECG signal to construct the classifier [29]. Due to the time-consuming nature of manual feature extraction and the low sensitivity of S, it has been difficult to meet the current demand for real-time classification of arrhythmia. Jinghao Niu (2020) used input data as a combination of raw heartbeat and RR interval features. To improve the classification performance of the classifier, Jinghao Niu (2020) used SBCX for the input heartbeats [41]. The accuracy of this article's method is lower than that of Jinghao Niu (2020) (91.89 to 95.87%), and the sensitivity of N is lower than that of Jinghao Niu (2020) (93.15% to 98.28%). However, the sensitivity of S is higher (80.23% to 77.35%) and the sensitivity of V is higher than that (90.99% to 85.08%) for the algorithm in this article. We compared our data input with that of Jinghao Niu (2020). The input data taken in this article is 508 points of raw heartbeats and is not filtered or preprocessed in any way. The input data taken in Jinghao Niu (2020) is a combination of 256 heartbeats and RR interval features and is preprocessed using SBCX. Therefore, the method proposed in this article is more automated.

The article "A Deep Neural Network Ensemble Classifier with Focal Loss for Automatic Arrhythmia Classification" was published in 2022. Journal: J Healthc Eng.

### 3.3. Ablation Studies

We conduct ablation studies on the different components of the framework. In Table 9, signal-508 represents the heartbeat segmentation method proposed in this article. Signal-256 represents the conventional 256-sample heartbeat segmentation method [41, 44]. Focal loss represents the loss function used in this article. Ensemble represents the model ensemble module.

Replacing the heartbeat segmentation method with the traditional 256-sample heartbeat segmentation method, the sensitivity of S is greatly reduced (80.23% to 16.34%), and the ability to classify S is almost lost. This fact strongly suggests that the heartbeat segmentation approach adopted in this article helps to improve the model's ability to classify heartbeats. The medical diagnosis of arrhythmia is not only based on a single heartbeat but is determined by combining multiple consecutive heartbeats. For example, S will have a shorter RR interval relative to N. When the heartbeat segmentation approach in this article is used, it helps to make it easier for the classifier to obtain distinct features to distinguish between N and S, preventing the overfitting of S during training. By replacing the focal loss with the traditional cross-entropy loss function, the sensitivity of S will decrease (80.23% to 61.60%). The focal loss function helps to make the model focus more on the hard-to-discriminate categories during training, and S, as the generally less sensitive type among the classification results of the various methods, is more likely to receive attention. After removing the ensemble module, the sensitivity of N decreased by 3.78% (93.15% to 89.37%), and that of S decreased by 8.61% (80.23% to 71.62%). In this research, six basic classifiers are trained for voting, resulting in a more robust classification model with increased performance. The comparisons in Table 9 demonstrate the effectiveness of our strategy.

## 4. Conclusion

This article proposes a brand-new system for classifying arrhythmias. In order to achieve a more automatic classification effect, we use the original heartbeat signal as the data input in this article. Three key characteristics define the classification model put forth in this article. First, we employ a novel heartbeat segmentation strategy to assist the model in automatically extracting more features. Second, in order to aid in model training, we use the focal loss as the loss function. Finally, an ensemble classifier is used to produce more reliable classification results. According to the analysis of the experimental data, increasing the input heartbeat window length enhances the model's classification performance, particularly in terms of its sensitivity to S. In the meantime, the ensemble training strategy used aids in reducing the issue of training overfitting brought on by data imbalance.

The article "A Deep Neural Network Ensemble Classifier with Focal Loss for Automatic Arrhythmia Classification" was published in 2022. Journal: J Healthc Eng.

The classification method proposed in this article is still plagued by low classification performance for *F* and *Q*. This is due to the fact that the *F* and *Q* samples in the MIT-BIH dataset are far too minimal. As a result, we intend to collect some additional arrhythmia data to help us better train the classification model in future work.

## Figures and Tables

**Figure 1:** Overall system structure diagram.

**Figure 2:** Diagram of the heartbeat segmentation strategy. (a) The traditional heartbeat segmentation strategy. (b) The heartbeat segmentation strategy proposed in this article. (c)(i) N by the traditional heartbeat segmentation strategy. c(ii) N by the segmentation strategy in this article. c(iii) S by the traditional heartbeat segmentation strategy. c(iv) S by the segmentation strategy in this article.

**Figure 3:** Overall structure of the classification algorithm.

**Figure 4:** Network structure of the base classifier.

**Table 1:** AAMI classification of heartbeat types.

Class	Symbol	Members
Normal	*N*	Normal beat left bundle branch block beat right bundle branch block beat atrial escape beat nodal (junctional) escape beat
Supraventricular ectopic beat	SVEB (*S*)	Atrial premature beat aberrated atrial premature beat nodal (junctional) premature beat supraventricular premature beat
Ventricular ectopic beat	VEB (*V*)	Premature ventricular contraction ventricular escape beat
Fusion beat	*F*	Fusion of ventricular and normal beat
Unknown beat	*Q*	Paced beat fusion of paced and normal beat unclassifiable beat

**Table 2:** Using interpatient division of training set DS1 and test set DS2.

Dataset	Patient numbers in the MIT-BIH arrhythmia database
DS1	101, 106, 108, 109, 112, 114, 115, 116, 118, 119, 122, 124, 201, 203, 205, 207, 208, 209, 215, 220, 223, 230
DS2	100, 103, 105, 111, 113, 117, 121, 123, 200, 202, 210, 212, 213, 214, 219, 221, 222, 228, 231, 232, 233, 234

**Table 3:** Heartbeat segmentation length and S sensitivity for different methods.

Work	Length of heartbeat	Sen (%) of S	Manually extracted features
Garcia (2017)	270	61.96	No
Takalo-mattila (2018)	130	62.49	No
Jinghao Niu (2020)	256	77.35/38.7	Yes/No
Haojie Zhang (2021)	256	88.24/8.06	Yes/No

**Table 4:** Proportion of each class of heartbeats.

Segment	*N*	*S*	*V*	*F*	*Q*
DS1	45824	943	3785	414	8
DS2	44215	1836	3219	388	7

The article "A Deep Neural Network Ensemble Classifier with Focal Loss for Automatic Arrhythmia Classification" was published in 2022. Journal: J Healthc Eng.

**Table 5:** Performance metrics of six base classifiers and ensemble model

Work	Acc (%)	+P (%)	Sen (%)	Spe (%)
^#^1	88.71	49.03	77.66	90.68
^#^2	88.18	47.66	83.61	89.37
^#^3	88.60	48.81	88.36	89.78
^#^4	86.92	44.58	85.64	87.91
^#^5	89.80	52.36	84.96	91.23
^#^6	83.54	38.14	84.92	83.91
Average	87.63	46.76	84.19	88.81
Result	91.89	59.51	85.37	93.15

**Table 6:** Confusion matrix of the ensemble classifier.

Predicted label						
		*N*	*S*	*V*	*F*	*Q*
True label	*N*	41186	1427	535	1067	0
	*S*	317	1473	42	4	0
	*V*	133	68	2929	89	0
	*F*	310	14	15	49	0
	*Q*	3	0	4	0	0

**Table 7:** Classification performance results of our method and 6 advanced methods.

Work	Acc	Class (N)			Class (S)			Class (V)		
		Sen (%)	+P (%)	Spe (%)	Sen (%)	+P (%)	Spe (%)	Sen (%)	+P (%)	Spe (%)
DeChazal (2004)	85.88	99.16	86.86	94.00	38.53	75.94	95.35	81.59	77.74	98.78
Garcia (2017)	92.38	93.99	97.95	82.55	61.96	52.96	97.89	87.34	59.44	95.91
Takalo-mattila (2018)	89.91	91.89	97.00	76.83	62.49	55.86	98.11	89.23	50.85	94.02
Sellami (2019)	88.34	88.52	98.8	91.3	82.04	30.44	92.8	92.05	72.13	97.54
Jinghao Niu (2020)	95.87	98.28	97.39	78.69	77.35	73.29	98.92	85.08	91.75	99.47
Yuanlu Li (2021)	88.99	94.54	93.33	80.8	35.22	65.88	98.83	88.35	79.86	94.92
Our methods	91.89	93.15	98.18	86.00	80.23	49.40	96.85	90.99	83.09	98.72

**Table 8:** Overall model performance metrics for our method and 6 advanced methods.

	Acc (%)	+P (%)	Sen (%)	Spe (%)
DeChazal (2004)	85.88	42.21	92.85	86.86
Garcia (2017)	92.38	59.36	81.73	93.99
Takalo-mattila (2018)	89.91	52.86	76.18	91.89
Sellami (2019)	88.34	48.25	90.90	88.51
Jinghao Niu (2020)	95.87	84.55	78.18	98.28
Yuanlu Li (2021)	88.99	56.82	52.10	94.75
Our methods	91.89	59.51	85.37	93.15

**Table 9:** Ablation studies on our proposed model.

Work	Acc (%)	Class (N)			Class (S)			Class (V)			Class (F)		
		Sen (%)	+P (%)	Spe (%)	Sen (%)	+P (%)	Spe (%)	Sen (%)	+P (%)	Spe (%)	Sen (%)	+P (%)	Spe (%)
Signal-256 + focal loss + Ensemble	89.52	93.63	95.39	63.25	16.34	14.60	96.33	85.15	77.32	98.27	5.41	3.17	98.70
Signal-508 + ensemble	88.34	93.62	97.66	81.80	61.60	40.79	96.57	89.00	84.94	98.91	4.90	1.67	97.74
Signal-508 + focal loss	88.18	89.37	97.92	84.61	71.62	33.87	94.63	90.71	69.81	97.28	11.86	3.69	97.56
Signal-508 + focal loss + ensemble	91.89	93.15	98.18	86.00	80.23	49.40	96.85	90.99	83.09	98.72	12.63	4.05	97.65

## Data Availability

The data used to support the findings of this study are included within the article.

## References

[1] AlGhatrif M., Lindsay J. (2012). A brief review: history to understand fundamentals of electrocardiography. *Journal of Community Hospital Internal Medicine Perspectives*.

The article "A Deep Neural Network Ensemble Classifier with Focal Loss for Automatic Arrhythmia Classification" was published in 2022. Journal: J Healthc Eng.

[2] Gaziano T. A., Bitton A., Anand S., Abrahams-Gessel S., Murphy A. (Feb 2010). Growing epidemic of coronary heart disease in low- and middle-income countries. *Current Problems in Cardiology*.

[3] Guler I., Ubeyli E. D. (2005). ECG beat classifier designed by combined neural network model. *Pattern Recognition*.

[4] Homaeinezhad M. R., Atyabi S. A., Tavakkoli E., Toosi H. N., Ghaffari A., Ebrahimpour R. (2012). ECG arrhythmia recognition via a neuro-SVM-KNN hybrid classifier with virtual QRS image-based geometrical features. *Expert Systems with Applications*.

[5] Luz E. J. d. S., Schwartz W. R., Camara-Chavez G., Menotti D. (2016). ECG-based heartbeat classification for arrhythmia detection: a survey. *Computer Methods and Programs in Biomedicine*.

[6] Yu S.-N., Chen Y.-H. (2007). Electrocardiogram beat classification based on wavelet transformation and probabilistic neural network. *Pattern Recognition Letters*.

[7] Ghaffari A., Homaeinezhad M. R., Akraminia M., Atarod M., Daevaeiha M. (2009). A robust wavelet-based multi-lead electrocardiogram delineation algorithm. *Medical Engineering & Physics*.

[8] Khorrami H., Moavenian M. (2010). A comparative study of DWT, CWT and DCT transformations in ECG arrhythmias classification. *Expert Systems with Applications*.

[9] Ye C., Coimbra M. T., Kumar B. V. K. V., Ieee Arrhythmia detection and classification using morphological and dynamic features of ECG signals.

[10] Kutlu Y., Kuntalp D. (2012). Feature extraction for ECG heartbeats using higher order statistics of WPD coefficients. *Computer Methods and Programs in Biomedicine*.

[11] Ye C., Kumar B. V. K. V., Coimbra M. T. (2012). Heartbeat classification using morphological and dynamic features of ECG signals. *IEEE Transactions on Biomedical Engineering*.

[12] Huang G.-B. (2014). An insight into extreme learning machines: random neurons, random features and kernels. *Cognitive Computation*.

[13] Zhang Z., Dong J., Luo X., Choi K.-S., Wu X. (2014). Heartbeat classification using disease-specific feature selection. *Computers in Biology and Medicine*.

[14] Elhaj F. A., Salim N., Harris A. R., Swee T. T., Ahmed T. (2016). Arrhythmia recognition and classification using combined linear and nonlinear features of ECG signals. *Computer Methods and Programs in Biomedicine*.

[15] Luz E., Menotti D., Ieee How the choice of samples for building arrhythmia classifiers impact their performances.

[16] de Lannoy G., Francois D., Delbeke J., Verleysen M. (2012). Weighted conditional random fields for supervised interpatient heartbeat classification. *IEEE Transactions on Biomedical Engineering*.

[17] Huang H., Liu J., Zhu Q., Wang R., Hu G. (2014). A new hierarchical method for inter-patient heartbeat classification using random projections and RR intervals. *BioMedical Engineering Online*.

The article "A Deep Neural Network Ensemble Classifier with Focal Loss for Automatic Arrhythmia Classification" was published in 2022. Journal: J Healthc Eng.

[18] Rahhal M. M. A., Bazi Y., Alajlan N. (2015). Classification of AAMI heartbeat classes with an interactive ELM ensemble learning approach. *Biomedical Signal Processing and Control*.

[19] Song M. H., Lee J., Cho S. P., Lee K. J., Yoo S. K. (2005). Support vector machine based arrhythmia classification using reduced features. *International Journal of Control, Automation and Systems*.

[20] Asl B. M., Setarehdan S. K., Mohebbi M. (2008). Support vector machine-based arrhythmia classification using reduced features of heart rate variability signal. *Artificial Intelligence in Medicine*.

[21] de Lannoy G., Francois D., Delbeke J., Verleysen M. Weighted SVMs and feature relevance assessment in supervised heart beat classification.

[22] Karpagachelvi S., Arthanari M., Sivakumar M. (2012). Classification of electrocardiogram signals with support vector machines and extreme learning machine. *Neural Computing & Applications*.

[23] Reddy G. T., Reddy M. P. K., Lakshmanna K., Rajput D. S., Kaluri R., Srivastava G. (2020). Hybrid genetic algorithm and a fuzzy logic classifier for heart disease diagnosis. *Evolutionary Intelligence*.

[24] Comert Z., Kocamaz A. F., Gungor S., Ieee Classification and comparison of cardiotocography signals with artificial neural network and extreme learning machine.

[25] Acharya U. R., Fujita H., Lih O. S., Hagiwara Y., Tan J. H., Adam M. (2017). Automated detection of arrhythmias using different intervals of tachycardia ECG segments with convolutional neural network. *Information Sciences*.

[26] Elhaj F. A., Salim N., Ahmed T., Harris A. R., Swee T. T. Hybrid classification of Bayesian and Extreme Learning Machine for heartbeat classification of arrhythmia detection.

[27] Golrizkhatami Z., Acan A. (2018). ECG classification using three-level fusion of different feature descriptors. *Expert Systems with Applications*.

[28] Guo L., Sim G., Matuszewski B. (2019). Inter-patient ECG classification with convolutional and recurrent neural networks. *Biocybernetics and Biomedical Engineering*.

[29] de Chazal P., O’Dwyer M., Reilly R. B. (2004). Automatic classification of heartbeats using ECG morphology and heartbeat interval features. *IEEE Transactions on Biomedical Engineering*.

[30] Shi H., Wang H., Huang Y., Zhao L., Qin C., Liu C. (2019). A hierarchical method based on weighted extreme gradient boosting in ECG heartbeat classification. *Computer Methods and Programs in Biomedicine*.

[31] Dias F. M., Monteiro H. L. M., Cabral T. W., Naji R., Kuehni M., Luz E. J. d. S. (2021). Arrhythmia classification from single-lead ECG signals using the inter-patient paradigm. *Computer Methods and Programs in Biomedicine*.

The article "A Deep Neural Network Ensemble Classifier with Focal Loss for Automatic Arrhythmia Classification" was published in 2022. Journal: J Healthc Eng.

[32] Yang P., Wang D., Zhao W.-B., Fu L.-H., Du J.-L., Su H. (2021). Ensemble of kernel extreme learning machine based random forest classifiers for automatic heartbeat classification. *Biomedical Signal Processing and Control*.

[33] Acharya U. R., Oh S. L., Hagiwara Y. (2017). A deep convolutional neural network model to classify heartbeats. *Computers in Biology and Medicine*.

[34] Li Y., Pang Y., Wang J., Li X. (2018). Patient-specific ECG classification by deeper CNN from generic to dedicated. *Neurocomputing*.

[35] Namburu A., Sumathi D., Raut R. (2022). FPGA-based deep learning models for analysing corona using chest X-ray images. *Mobile Information Systems*.

[36] Garcia G., Moreira G., Menotti D., Luz E. (2017). Inter-patient ECG heartbeat classification with temporal VCG optimized by PSO. *Scientific Reports*.

[37] Takalo-Mattila J., Kiljander J., Soininen J.-P. Inter-patient ECG classification using deep convolutional neural networks.

[38] Han B., Jhaveri R., Wang H., Qiao D., Du J. (2021). Application of robust zero-watermarking scheme based on federated learning for securing the healthcare data. *IEEE journal of biomedical and health informatics*.

[39] Li Y., Qian R., Li K. (2022). Inter-patient arrhythmia classification with improved deep residual convolutional neural network. *Computer Methods and Programs in Biomedicine*.

[40] Sellami A., Hwang H. (2019). A robust deep convolutional neural network with batch-weighted loss for heartbeat classification. *Expert Systems with Applications*.

[41] Niu J. H., Tang Y. Q., Sun Z. Y., Zhang W. S. (2020). Inter-patient ECG classification with symbolic representations and multi-perspective convolutional neural networks. *Ieee Journal of Biomedical and Health Informatics*.

[42] Moody G. A., Mark R. G. (2001). The impact of the MIT-BIH arrhythmia database. *IEEE Engineering in Medicine and Biology Magazine*.

[43] Chawla N. V., Bowyer K. W., Hall L. O., Kegelmeyer W. P. (2002). SMOTE: synthetic minority over-sampling technique. *Journal of Artificial Intelligence Research*.

[44] Zhang H. J., Yang G. P., Huang Y. W., Yuan F., Yin Y. L. Multi-scale and attention based ResNet for heartbeat classification. *International Conference on Pattern Recognition*.

[45] Webb G. I., Zheng Z. J. (2004). Multistrategy ensemble learning: reducing error by combining ensemble learning techniques. *IEEE Transactions on Knowledge and Data Engineering*.

[46] Breiman L. (2001). Random forests. *Machine Learning*.

[47] Lin T.-Y., Goyal P., Girshick R., He K., Dollar P. (2020). Focal loss for dense object detection. *IEEE Transactions on Pattern Analysis and Machine Intelligence*.

The article "A Deep Neural Network Ensemble Classifier with Focal Loss for Automatic Arrhythmia Classification" was published in 2022. Journal: J Healthc Eng.

[48] Ioffe S., Szegedy C. Batch normalization: accelerating deep network training by reducing internal covariate shift.

[49] Srivastava N., Hinton G., Krizhevsky A., Sutskever I., Salakhutdinov R. (2014). Dropout: a simple way to prevent neural networks from overfitting. *Journal of Machine Learning Research*.

[50] He K., Zhang X., Ren S., Sun J., Ieee Deep residual learning for image recognition.

